# Efficacy of Laparoscopic Totally Extraperitoneal Repair for Inguinal Hernia

This article has been retracted.

**DOI:** 10.1155/2022/2970257

**Published:** 2022-09-24

**Authors:** Zhigang Pan, Minjie Zhang, Ling Wang

**Affiliations:** ^1^Director's Office, Jingxian Hospital of Anhui Province, Xuancheng, China; ^2^Department of Surgical, Jingxian Hospital of Anhui Province, Xuancheng, China; ^3^Office, Jingxian Hospital of Anhui Province, Xuancheng, China

## Abstract

**Objective:**

To assess the treatment efficacy of laparoscopic totally extraperitoneal repair for inguinal hernia.

**Methods:**

Between November 2018 and May 2020, 130 patients with inguinal hernias diagnosed and treated in our hospital were randomly recruited and assigned to receive either tension-free hernia repair (control group) or laparoscopic totally extraperitoneal repair (study group) at the random method. All patients received routine care including external traditional Chinese medicine (TCM) application. Outcome measures included surgical indices, numeric rating scale (NRS) scores, infections, and postoperative complications.

**Results:**

Laparoscopic surgery is associated with a shorter operation duration, time-lapse before postoperative off-bed activity, and hospital stay, as well as less intraoperative hemorrhage volume compared to tension-free hernia repair in the control group. Patients in the study group had considerably lower NRS ratings after therapy than those in the control group. (*P* < 0.05). After treatment, the levels of blood cell count (WBC), C-reactive protein (CRP), and procalcitonin (PCT) in the study group were lower than those in the control group (*P* < 0.05). In the control group, there were 0 cases of hematoma, 3 cases of subcutaneous effusion, 4 cases of urinary retention, 5 cases of scrotal effusion, and 1 case of bladder injury. In the study group, there were 0 cases of hematoma, 1 case of subcutaneous fluid, 1 case of urinary retention, 0 cases of scrotal fluid, and 0 cases of bladder injury. Laparoscopic surgery resulted in a lower incidence of postoperative complications versus traditional surgery (*P* <0.05).

**Conclusion:**

Laparoscopic totally extraperitoneal repair for inguinal hernia improves the intraoperative indices, mitigates postoperative pain, and reduces the risks of infections and complications, with the advantages of short operation duration, less hemorrhage volume, and shorter hospital stay. It shows great potential for clinical promotion.

## 1. Introduction

Inguinal hernia [1] refers to the dislocation of an organ or tissue in the body. The inguinal region is a triangular area with the thigh as the lower limit, the lateral edge of the abdomen as the inner edge, and the horizontal line between the upper foreskin and the lateral edge of the abdomen as the upper limit [2, 3]. Despite the unclear etiology, the associated epidemiology suggests that an inguinal hernia is primarily associated with abdominal wall weakness and increased intra-abdominal pressure. According to the recommendations for the treatment of inguinal hernia in adults, more than 20 million inguinal operations are performed globally each year [4], with an incidence of 1-5% in the elderly over 60 years of age and a male to female incidence ratio of 15 : 1. There are various causes for the disease onset, such as dysplasia of the groin, aging, poor growth, malnutrition, abdominal metabolism, or previous lower abdominal surgery [5].

Inguinal hernias are divided into indirect hernias and direct hernias [6]. Indirect hernias protrude from the deep ring of the inguinal passage, which is located on the side of the inferior epigastric artery, and travel inward and downward, obliquely through the inguinal passage, and then through the superficial inguinal ring, reaching the scrotum, accounting for approximately 95% of all inguinal hernias. Direct hernias protrude directly posteriorly from the inguinal triangle within the inferior epigastric artery, without crossing the internal ring nor reaching the scrotum, and account for only 5% of inguinal hernias [7, 8]. Untimely interventions may lead to serious complications that pose a serious threat to the patient's health. Clinical treatment of inguinal hernia includes conservative treatment and surgical treatment. However, conservative treatment fails to deliver consistently favorable efficacy, and surgical therapy is mostly adopted.

Tension-free hernioplasty (OTFH) [9] is the standard procedure for effective treatment, but recent clinical data show that it has many postoperative complications and a high recurrence rate [10]. Laparoscopic totally extraperitoneal prosthesis (TEP) [11] is a novel procedure first proposed by McKernan et al. in 1992 [12]. It is performed through a subumbilical preperitoneal approach to release the preperitoneal space, remove the hernia sac from the spermatic cord peritonealization, and place an extraperitoneal patch to repair the pubococcygeal muscle foramen. Compared to tension-free hernia repair, this procedure obviates the need for the opening of the patient's abdominal cavity and allows for a direct operation on the patient's anterior peritoneal space to complete the treatment, with benefits such as less pain, faster recovery, and a lower risk of complication [13, 14]. Nevertheless, the laparoscopic totally extraperitoneal prosthesis is demanding for the surgeon, and its efficacy varies depending on the surgeon's skill. Here, the present study was undertaken to assess the treatment efficacy of laparoscopic totally extraperitoneal repair for inguinal hernia.

## 2. Materials and Methods

### 2.1. Participants

Totally 130 patients (104 males and 26 females, aged between 20–75 years) with inguinal hernia diagnosed and treated in our hospital between November 2018 and May 2020 were randomly recruited and assigned to receive either traditional treatment, i.e., tension-free hernia repair (control group) or laparoscopic totally extraperitoneal repair (study group) alternately at the point of admission order. The randomization was carried out using an online web-based randomization tool (freely available at http://www.randomizer.org/). For concealment of allocation, the randomization procedure and assignment were managed by an independent research assistant who was not involved in the screening or evaluation of the participants.

#### 2.1.1. Sample Size Estimation

The original sample size calculation estimated that 60 patients in each group would be needed to detect a 3-point difference between groups in a 2-sided significance test with a power of 0.8 and an alpha error level of 0.05.

#### 2.1.2. Ethical Considerations

The study protocol and all amendments were approved by the appropriate ethics committee at each centre. The study was done in accordance with the protocol, its amendments, and standards of clinical practice. All participants provided written informed consent before enrolment. Ethics no.: YU-TY20180102.

### 2.2. Inclusion and Exclusion Criteria

Inclusion criteria: patients who met the relevant diagnostic criteria of inguinal hernia, with consciousness and normal communication ability, without mental illness, and who provided written informed consent were included.

Exclusion criteria: patients with serious dysfunction of heart, lung, liver, and kidney, with abdominal surgery within the last six months and with contraindications to surgery were excluded.

### 2.3. Treatment

Patients in the control group were treated with tension-free hernia repair. The patient was given continuous epidural anesthesia, a 5 cm incision was made parallel to the groin, the external oblique tendon membrane and levator muscle were incised, the location of the hernia pouch was determined, and the hernia treatment belt was tied. After patch trimming, the hernia belt was properly placed, the combined osteochondral and ligamentous dressings and ligaments were fixed with sutures and bandages, and the lumbar belt was compressed 24 hours postoperatively.

Patients in the study group received laparoscopic totally extraperitoneal repair. Anesthesia and tracheal intubation were done with the patient in the Trendelenburg position. The anterior abdominal sheath was incised, and an incision was created for intubation. Trocars were placed in the middle, higher, and 1/3 middle of the line between the pubic bone and the umbilicus, and the spermatic cord and internal annulus were isolated from other critical structures as well as the vas deferens, hernia sac, and spermatic arteries. The patch was placed, the peritoneum was naturally repositioned, the trocar was removed, and the abdominal wall was sutured.

All patients received routine care including external traditional Chinese medicine (TCM) application. 200 g of Natrii Sulfas and 50 g of borneolum syntheticum were powdered, mixed thoroughly, and then packed in a cloth bag sewn with a cotton cloth and sealed. It was administered externally to the inguinal and scrotal regions on the operated side after surgery: the incision was covered with two layers of sterile gauze, the cotton bag was uniformly put on the sterile gauze and sealed with adhesive tape, and the topical pack was replaced once daily. If the patient experienced localized skin redness or other serious adverse reactions, the topical application was stopped immediately.

### 2.4. Outcome Measures

1. Surgical condition: the surgical condition of patients in both groups was recorded, including operation time, intraoperative bleeding, time-lapse before postoperative off-bed activity, and length of hospital stay
2. Pain score: the patients' pain was evaluated with reference to the numeric rating scale (NRS) score, and the scale has a total score of 10 points, with 0 points for no pain, 1-3 points for mild pain, 4-6 points for moderate pain, and 7-10 points for severe pain. The score was proportional to the severity of the pain
3. Infectious indices: 5 ml of fasting venous blood was collected from all patients, placed in a dry tube, and centrifuged at 3500 r/min for 15 min, and the serum was separated for the determination of white blood cell count (WBC), C-reactive protein (CRP), and procalcitonin (PCT) using a Beckman hematocrit analyzer (model: DxH 600, Shilian Boyan Beijing Technology Co. (PCT).
4. Complications: the occurrence of complications, including hematoma, subcutaneous effusion, urinary retention, scrotal effusion, and bladder injury, were recorded

### 2.5. Statistical Analysis

The mean difference between the two groups was tested using student's *t*-test for normally distributed variables and Mann–Whitney U test for non-normal variables. SPSS 22.0 software was used for data analyses. Measurement data are expressed as (mean ± standard deviation) and analyzed using the independent sample *t*-test. Count data are expressed as frequency (%) and analyzed using the chi-square test. *P* < 0.05 was set as a cut off for statistical significance.

## 3. Results

### 3.1. Patient Characteristics

In the control group, there were 65 patients, 53 males and 12 females, aged 25-69 (40.35 ± 7.28) years, with a mean BMI of 21.98 ± 2.17 kg/m2. There were 20 cases of bilateral hernia, 45 cases of unilateral hernia, 24 cases of direct hernia, and 41 cases of indirect hernia. In the study group, there were 65 patients, 51 males and 14 females, aged 23-68 (40.85 ± 6.99) years, with a mean BMI of 22.03 ± 2.21 kg/m^2^. There were 22 cases of bilateral hernia, 43 cases of unilateral hernia, 20 cases of direct hernia, and 45 cases of indirect hernia. The patient characteristics between the two groups were comparable (*P* > 0.05) (Table 1).

### 3.2. Surgical Indices

Laparoscopic surgery was associated with a shorter operation length, time-lapse before postoperative off-bed activities, and hospital stay as well as decreased intraoperative bleeding volume, compared to conventional surgery in the control group. (*P* < 0.05) (Table 2).

### 3.3. NRS Scores

Before treatment, there were no significant differences in the NRS scores between the two groups (*P* > 0.05). After treatment, patients in the study group had significantly lower NRS scores (2.95 ± 0.98) than those in the control group (4.87 ± 1.04) (*P* < 0.05) (Table 3).

### 3.4. Infectious Indices

Before treatment, the two groups of patients showed similar levels of WBC, CRP, and PCT (*P* > 0.05). After treatment, the levels of WBC, CRP, and PCT in the study group were lower than those in the control group (*P* < 0.05) (Table 4).

### 3.5. Postoperative Complications

In the control group, there were 0 (0.00%) cases of hematoma, 3 (4.62%) cases of subcutaneous effusion, 4 (6.15%) cases of urinary retention, 5 (7.69%) cases of scrotal effusion, and 1 (1.54%) case of bladder injury. In the study group, there were 0 (0.00%) cases of hematoma, 1 (1.54%) case of subcutaneous fluid, 1 (1.54%) case of urinary retention, 0 (0.00%) cases of scrotal fluid, and 0 (0.00%) cases of bladder injury. Laparoscopic surgery resulted in a lower incidence of postoperative complications (3.08%) versus traditional surgery (20.00%) (*P* < 0.05) (Table 5).

## 4. Discussion

Inguinal hernia is a common surgical condition [15], which, if left untreated, predisposes to ischemia and necrosis of the intestinal cavity or other abdominal areas. Aside from hernias in infants, the disease commonly requires surgical repair [16]. The first classical hernia repair used sutures on both sides of the lesion, but it was associated with high surgical wound tension, postoperative pain, and a high recurrence rate. Thus, it was gradually replaced by tension-free hernia repair to reduce the risk of disease recurrence. [17]. In recent years, with the improvement of medical technology, laparoscopic inguinal hernia repair has been gradually adopted. Laparoscopic total extraperitoneal hernia repair is a laparoscopic repair of an anterior peritoneal hernia performed in the posterior approach without operating inside the patient's abdominal cavity, resulting in minimal surgical trauma and rapid postoperative wound healing. In view of this, a total of 130 patients with inguinal hernia diagnosed and treated in our hospital were recruited to assess the treatment efficacy of laparoscopic totally extraperitoneal repair for inguinal hernia.

The results showed that laparoscopic totally extraperitoneal repair was associated with shorter operation duration, time-lapse before postoperative off-bed activity, and hospital stay, and less intraoperative hemorrhage volume (*P* < 0.05), indicating that the laparoscopic surgery had a shorter operation duration, less intraoperative hemorrhage, and better postoperative recovery. The reason may be that the laparoscopic totally extraperitoneal repair [18] is less traumatic and benefits the patients' postoperative recovery, thereby shortening the treatment course and promoting their early recovery. In addition, patients in the study group showed significantly lower NRS scores than those in the control group (*P* < 0.05). The reason may be that laparoscopic total extraperitoneal hernia repair expands the surgical field of view and improves the accuracy and effectiveness of surgical operation to avoid damage to surrounding tissues and organs. In addition, it avoids excessive separation of the triangle of doom, and the placement of the patch is more in line with the physiological anatomy of the human body, allowing tension-free repair of the defect. Secondly, this surgical approach eliminates the need for fixed mesh and results in less postoperative pain, shorter time to get out of bed and shorter hospital stay for the patient due to less damage to normal tissues [19, 20]. The small trauma of laparoscopy and the use of general anesthesia [21] alleviate patient pain and prevent pain-induced stress reactions to relieve patient pain, which is consistent with the findings of Sanna et al.

Laparoscopic surgery herein resulted in lower levels of WBC, CRP, and PCT versus tension-free surgery (*P* < 0.05). Leukocytes absorb foreign substances to create antibodies and inhibit pathogen invasion. Leukocyte counts may be pathologically elevated under the influence of the groin as a result of surgical trauma, which is useful in determining the existence of inflammation [22]. C-reactive protein is an acute phase protein that significantly increases in the body when there is an infection or tissue damage. C-reactive protein levels typically rise after surgery and fall one week later, with the absence of another fall or rise indicating a potential risk of infection or thromboembolism [23, 24]. PCT reflects the active degree of the inflammatory response of the body, and its variations contribute to the timely adjustment of the treatment plan. Based on the above results, it is reasonable to conclude that the use of laparoscopic totally extraperitoneal repair for inguinal hernia effectively reduces the risk of postoperative infection in patients, which is consistent with the results. Moreover, the overall incidence of complications was significantly lower in the study group (3.08%) than in the control group (20.00%) (*P* < 0.05).

Notably, the complications in both groups were better than in previous similar studies, which was attributed to the addition of TCM application after surgery. The main clinical methods for mitigating scrotal seroma are local compression and intraoperative placement of drainage, but the clinical outcomes are mediocre. TCM external application is to allow absorption of effective drug ingredients into the body through human arteries, skin stratum corneum, and deep epidermis. Natrii Sulfas is a TCM herb that has the effect of softening the hardness and diarrhea, clearing heat and dampness, and reducing swelling and analgesia. Natrii Sulfas may induce constriction of local blood vessels and reduce incisions and swelling, and laparoscopic surgery results in a low risk of local tissue injury and obviates the need for suturing the peritoneum, significantly lowering the risk of complications after abdominal surgery [25]. However, laparoscopic totally extraperitoneal inguinal hernia repair requires a high requirement for the surgeons, and the anatomical structures are usually difficult to identify, especially in patients with severe adhesions or large cysts.

In this study, based on the disease characteristics of inguinal hernia patients, laparoscopic total extraperitoneal hernia patch repair was performed to provide insights for future postoperative treatment and to suggest the feasibility of external compression of traditional Chinese medicine. This study has the following limitations: (1) The sample size of this trial was small, and the significant differences in postoperative efficacy between the two groups could not be evaluated more comprehensively and objectively from the perspective of a large sample size. (2) The study used more subjective efficacy assessment criteria, and it is difficult to provide an absolutely objective and accurate description of the assessment on the scale due to the large differences in subjective perceptions among individuals, different cultural levels, and differences in the understanding of the questions in the scale. (3) This trial has a short postoperative follow-up period, and the long-term therapeutic effects were not observed. (4) This study lacks animal testing to clarify the drug targets on which the combination of these three drugs is based, resulting in a lack of a scientific basis.

## 5. Conclusion

Laparoscopic totally extraperitoneal repair for inguinal hernia improves the intraoperative indices, mitigates postoperative pain, and reduces the risks of infections and complications, with the advantages of short operation duration, less hemorrhage volume, and shorter hospital stay. It shows great potential for clinical promotion.

## Figures and Tables

**Table 1:** Patient characteristics ($\bar{x}\pm s$).

Group	*n*	Range		Age (year)		BMI (kg/m^2^)	Pathological types			
		Male	Female	Range	Mean		Bilateral hernia	Unilateral hernia	Direct hernia	Indirect hernia
Control	65	53	12	25-69	40.35 ± 7.28	21.98 ± 2.17	20	45	24	41
Study	65	51	14	23-68	40.85 ± 6.99	22.03 ± 2.21	22	43	20	45
*t*	—	—	—	—	0.399	0.130	—	—	—	—
*P* value	—	—	—	—	0.691	0.897	—	—	—	—

**Table 2:** Surgical indices ($\bar{x}\pm s$).

Group	*n*	Operation duration (min)	Intraoperative hemorrhage volume (ml)	Time-lapse before postoperative off-bed activity (h)	Hospital stay (d)
Control	65	69.15 ± 20.18	32.54 ± 12.35	70.08 ± 6.72	7.78 ± 2.98
Study	65	56.17 ± 12.35	25.15 ± 8.87	25.24 ± 3.68	4.15 ± 1.21
*t*	—	12.851	6.053	35.459	4.987
*P* value	—	<0.001	<0.001	<0.001	<0.001

**Table 3:** NRS scores ($\bar{x}\pm s$).

Group	*n*	Before treatment	After treatment
Control	65	6.85 ± 1.85	4.87 ± 1.04
Study	65	6.79 ± 2.01	2.95 ± 0.98
*t*	—	0.415	3.377
*P* value	—	0.657	<0.001

Note: ^∗^indicates statistically significant differences (*P* < 0.05) between pre- and posttreatment results in the same group of patients.

**Table 4:** Infectious indices ($\bar{x}+s$).

Timepoint	Indices	Control (*n* = 65)	Study (*n* = 65)	*t*	*P* value
Before treatment	WBC (x10^9^/L)	6.11 ± 0.83	6.15 ± 0.80	0.325	0.738
	CRP (mg/L)	4.95 ± 0.15	4.98 ± 0.18	0.151	0.895
	PCT (ng/mL)	0.26 ± 0.07	0.25 ± 0.08	0.038	0.997

After treatment	WBC (x10^9^/L)	17.56 ± 2.08	14.88 ± 0.56	3.256	<0.001
	CRP (mg/L)	8.28 ± 1.56	6.25 ± 0.98	4.568	<0.001
	PCT (ng/mL)	0.55 ± 0.16	0.34 ± 0.10	5.687	<0.001

Note: ^∗^indicates statistically significant differences (*P* < 0.05) between pre- and posttreatment results in the same group of patients.

**Table 5:** Postoperative complications (%).

Group	*n*	Hematoma	Subcutaneous fluid	Urinary retention	Scrotal fluid	Bladder injury	Total incidence
Control	65	0 (0.00)	3 (4.62)	4 (6.15)	5 (7.69)	1 (1.54)	13 (20.00)
Study	65	0 (0.00)	1 (1.54)	1 (1.54)	0 (0.00)	0 (0.00)	2 (3.08)
*x* ^2^	—	4.598					
*P* value	—	0.031					

## Data Availability

All data generated or analysed during this study are included in this published article.
